The article "Salviae miltiorrhizae Liguspyragine Hydrochloride and Glucose Injection Protects against Myocardial Ischemia-Reperfusion Injury and Heart Failure" was retracted in 2023. Reasons: signs of a paper mill; suspected computer-generated content; unreliable results or conclusions; concerns about the data.

# Salviae miltiorrhizae Liguspyragine Hydrochloride and Glucose Injection Protects against Myocardial Ischemia-Reperfusion Injury and Heart Failure

**DOI:** 10.1155/2022/7809485

**Published:** 2022-06-29

**Authors:** Shang Kong, Dan Zhou, Qinghong Fan, Tingting Zhao, Chunguang Ren, Hong Nie

**Affiliations:** ^1^Guangdong Province Key Laboratory of Pharmacodynamic Constituents of TCM and New Drugs Research, College of Pharmacy, Jinan University, Guangzhou 510632, China; ^2^International Cooperative Laboratory of Traditional Chinese Medicine Modernization and Innovative Drug Development of Chinese Ministry of Education (MOE), College of Pharmacy, Jinan University, Guangzhou 510632, China; ^3^Laboratory of Developmental Biology, Department of Cell Biology and Genetics, Chongqing Medical University, Chongqing 400016, China

## Abstract

**Purpose:**

Myocardial ischemia-reperfusion (MIR) injury is a common stimulus for cardiac diseases like cardiac arrhythmias and heart failure and may cause high mortality rates. Salviae miltiorrhizae liguspyragine hydrochloride and glucose injection (SGI) has been widely used to treat myocardial and cerebral infarctions in China even though its pharmacological mechanisms are not completely clear.

**Methods:**

The protective effect and mechanism of SGI on MIR injury and heart failure were investigated through the H9c2 cell model induced by hypoxia/reoxygenation (H/R) and rapamycin, zebrafish model induced by H/R and isoprenaline, and rat MIR model.

**Results:**

SGI significantly reduced the infarct size and alleviated the impairment of cardiac functions in the MIR rat model and H/R zebrafish model and promoted cell viability of cardiomyocyte-like H9c2 cells under H/R condition. Consistently, SGI significantly downregulated the serum level of biomarkers for cardiac damage and attenuated the oxidative damage in the MIR and H/R models. We also found that SGI could downregulate the increased autophagy level in those MIR and H/R models since autophagy can contribute to the injurious effects of ischemia-reperfusion in the heart, suggesting that SGI may alleviate MIR injury via regulating the autophagy pathway. In addition, we demonstrated that SGI also played a protective role in the isoproterenol-induced zebrafish heart failure model, and SGI significantly downregulated the increased autophagy and SP1/GATA4 pathways.

**Conclusion:**

SGI may exert anti-MIR and heart failure by inhibiting activated autophagy and the SP1/GATA4 pathway.

## 1. Introduction

Cardiovascular diseases, mostly ischemic heart disease and stroke, are the leading cause of global mortality [1]. Myocardial ischemia-reperfusion (MIR) injury plays a critical role in the pathogenesis of ischemic heart disease [2, 3]. Myocardial tissue relies on blood perfusion to maintain normal function, metabolism, and morphological structure, and reduced coronary blood supply to the myocardium causes an insufficient supply of oxygen and nutrients resulting in myocardial ischemia (MI) [3, 4]. Although restoration of blood flow to an ischemic heart prevents irreversible myocardial tissue injury, reperfusion alone often causes more tissue damage than that is caused by ischemia, and this reperfusion-induced injury is known as MIR injury [5]. MIR injury is characterized by the structural, functional, and biochemical changes in the myocardial tissue and results in arrhythmia, infarct size enlargement, and persistent ventricular systolic dysfunction [6]. Many pathophysiological processes including ion accumulation, mitochondrial membrane damage, the formation of reactive oxygen species, disturbances in nitric oxide metabolism, endothelial dysfunction, platelet aggregation, immune activation, apoptosis, and autophagy are involved in MIR injury [7]. Importantly, autophagy plays differential roles in MI injury and reperfusion injury, respectively [8]. Activation of autophagy in cardiomyocytes has been shown to protect against ischemic damage through providing energy substrate, removing damaged mitochondria, and reducing oxidative stress [9, 10]. Autophagy activation during cardiac ischemia is triggered by activation of the AMPK pathway and inhibition of the Rheb/mTOR pathway, and disruption of these mechanisms impairs autophagy activation and exacerbates myocardial injury [11–14]. Additionally, hypoxia-induced autophagy has been shown to promote cardiomyocyte survival through the PI3K/AKT/mTOR pathway [15]. In contrast, autophagy is massively activated during reperfusion in Beclin1-dependent but AMPK-independent manners [11], and cardiac damage during ischemia-reperfusion can be protected by preventing excessive autophagy [16, 17].

The article "Salviae miltiorrhizae Liguspyragine Hydrochloride and Glucose Injection Protects against Myocardial Ischemia-Reperfusion Injury and Heart Failure" was retracted in 2023. Reasons: signs of a paper mill; suspected computer-generated content; unreliable results or conclusions; concerns about the data.

Heart failure is described by ventricular systolic or diastolic dysfunction associated with a high rate of mortality and morbidity [18], and the most common cause of heart failure is MI [19]. Before heart failure, patients usually show myocardial hypertrophy phenotype, which is a sign of heart remodeling. Increased autophagy activation appears in a variety of animal models of heart failure [20]. Atrial natriuretic peptide (ANP) and brain natriuretic peptide (BNP) are secreted by damaged cardiomyocytes and are widely used as important indicators for clinical diagnosis of heart failure and cardiac dysfunction [21, 22]. In terms of the pharmacological therapy of MIR injury, more than 20 drugs have shown certain clinical efficacy on MIR injury by targeting one or more pathophysiological processes including reactive oxygen species production, calcium increase, and inflammation [23]. Myocardial ischemia and heart failure are not completely different models, they are closely related, and long-term myocardial ischemia will lead to heart failure. Clinically, ischemic heart disease is one of the main causes of heart failure, and treatment of myocardial ischemia disease is closely related to the treatment of heart failure. However, a universally accepted treatment is still lacking, and it is necessary to continue the discovery of new therapeutic agents applied during reperfusion to protect the heart against ischemia-reperfusion damage.

Salivae miltiorrhizae liguspyragine hydrochloride and glucose injection (SGI) is an infusion dosage form consisting of Salvia miltiorrhiza extract and ligustrazine, with main acting substances represented by tanshinol and ligustrazine hydrochloride [24]. The SGI has been proved with a protective effect on the acute myocardial infarction rat model [25], and SGI was also reported to significantly improve the neurological deficit score in patients with acute cerebral infarction [26]. However, it is still unknown whether SGI plays therapeutic roles in other cardiovascular diseases like MIR injury and heart failure. We demonstrated the role of SGI in the prevention and alleviation of MIR injury and heart failure in the present study, and the molecular mechanism study showed that SGI may exert those effects via limiting the activation of the autophagy-related signal pathways and the natriuretic peptide pathway.

## 2. Material and Methods

### 2.1. Reagents and Antibodies

SGI was supplied by Guizhou Jingfeng Injection Co., Ltd. (Guiyang, China). Sulfotanshinone sodium injection (Tan IIA) was purchased from Shanghai No. 1 Biochemical Pharmaceutical Co., Ltd. (Shanghai, China). Isoproterenol (ISO) was obtained from Dalian Meilun Biotechnology Co., Ltd. (Dalian, China). The reagent information used in the experiment is provided in the supplementary material (Table S1).

### 2.2. Animals and Diets

Specific pathogen-free (SPF) male Sprague-Dawley rats (150-170 g, certificate: No. 44007200057938) were purchased from the Medical Laboratory Animal Research Center of Guangdong Province (No. SCXK (Yue) 2013-0002). All rats were housed in an SPF environment in the Institution of Laboratory Animal Science of Jinan University with normal temperature and 12 h light-dark cycle. Rats were provided with a standard laboratory diet and water. The experiments were approved by the Committee on Animal Care of Jinan University (No. IACVC-20180918-06) and were conducted according to the instructions of the Laboratory Animal Ethics Committee of Jinan University. See supplementary materials for other treatment methods.

The article "Salviae miltiorrhizae Liguspyragine Hydrochloride and Glucose Injection Protects against Myocardial Ischemia-Reperfusion Injury and Heart Failure" was retracted in 2023. Reasons: signs of a paper mill; suspected computer-generated content; unreliable results or conclusions; concerns about the data.

### 2.3. Determination of the Zebrafish Cardiac Function

To detect the heart function of zebrafish, the zebrafish embryos at 4 days post fertilization were placed at room temperature, and the heartbeat of 15 s was recorded under a microscope and multiplied by 4 to get the heartbeat for 1 minute [27]. For the imaging, we placed the zebrafish embryo in a Petri dish and fixed it with 1% low-melting agar to make it lie on its side. An inverted fluorescence microscope was used (Leica, Germany) to image continuously for 5 seconds to generate 58 pictures, and the diastolic and systolic pictures were selected and processed with the ImageJ to quantify the length (a) and width (b) of the ventricle. We calculated the zebrafish's stroke volume (SV), ejection fraction (EF), fractional area change (FAC), and cardiac output (CO). See the supplementary materials for the specific calculation formula.

### 2.4. Quantitative RT-PCR

Zebrafish RNA extraction, reverse transcription, and quantitative amplification were performed following the instructions of the kit obtained from Nanjing Vazyme Biotech Co., Ltd., and the article numbers are RC101, R223-01, and Q711-02. The primer sequence is shown in the supplementary material (Table S2). The data were processed using the 2^-*ΔΔ*Ct^ method for the calculation of relative gene expression [28–31].

### 2.5. Western Blot Analysis

Total proteins were extracted from heart tissues. Protein concentrations were determined by the BCA protein assay. Each sample containing 30 mg of protein was, respectively, separated into 8%, 10%, and 15% sodium dodecyl sulfate-polyacrylamide gel electrophoresis and transferred to a polyvinylidene difluoride membrane. Thereafter, the membranes were incubated in 5% (volume weight) milk solution for 2 h and then incubated overnight at 4°C. See the supplementary materials for other detailed procedures.

### 2.6. Immunofluorescent Analysis

Immunofluorescence was used to detect Beclin1 and LC-3 in myocardial tissue. The left ventricular tissues were frozen and sectioned, rewarmed at room temperature, air-dried, and fixed with paraformaldehyde for 10 min. After the paraformaldehyde was completely dried, the tissues were washed 3 times with PBS, shaken on a decolorizing shaker, and fixed for 5 min each time. See the supplementary materials for other detailed procedures.

### 2.7. Myocardial Tissue Structure Was Observed by Transmission Electron Microscopy

Myocardial tissue samples were collected and fixed with 2.5% glutaraldehyde solution at 4°C overnight. Then, the samples were treated as follows (see the supplementary material for the detailed process).

The article "Salviae miltiorrhizae Liguspyragine Hydrochloride and Glucose Injection Protects against Myocardial Ischemia-Reperfusion Injury and Heart Failure" was retracted in 2023. Reasons: signs of a paper mill; suspected computer-generated content; unreliable results or conclusions; concerns about the data.

### 2.8. Statistical Analysis

The experimental data were processed with SPSS 20.0 software, and one-way ANOVA was used to compare and analyze significant discrepancies between the groups. *P* < 0.05 indicates a statistically significant discrepancy. The experimental results are expressed as the means ± SEMs and analyzed using GraphPad Prism 6.

## 3. Results

### 3.1. SGI Reduces Myocardial Infarction Damage in a Rat MIR Model

To study the role of SGI treatment in MIR injury, we established a rat MIR injury model, in which the normal and infarct areas were colored in dark blue and red, respectively. Similar to the Tan IIA treatment group, which has been clinically widely used for treating coronary heart diseases and thus selected as the positive control, SGI treatments with multiple dosages all ameliorated ischemia-reperfusion injuries to the hearts by lessening ischemia-reperfusion-induced changes in infarction areas (Figures 1(a) and 1(b)). In addition, we also measured the heart rate and S-T segment among the treatment groups, and we observed a decrease in heart rate under ischemic conditions, although there was no significant difference between the SGI groups and other groups under the normal, ischemic, and reperfusion conditions (Figures 1(c) and S1a). Compared to the model group, the S-T segment of the SGI groups was significantly lower both under the reperfusion and ischemia conditions (Figures 1(d) and S1b). In addition, an electrocardiogram was monitored to predict the severity of ischemia-induced myocardial damage. And the S-T segment of the SGI group and Tan IIA group showed elevation during ischemia while decreasing during the reperfusion condition (Figure S1c). We further performed the transmission electron microscopy analysis of the fine details of the myocardial structure. The transmission electron microscopy analysis results showed a disordered arrangement of myocardial fibers, dissolution of myofilaments, the sonic velocity of mitochondria, and the presence of cytoplasmic vesicles that may represent autophagosomes in the model group (Figure 1(e)). And there was a significant improvement in the myocardial fibers' alignment and mitochondria shape in the SGI groups. Taken together, the above results indicated that SGI protects against MIR injury.

As a result of myocardial damage, many proteins and enzymes are released from the heart tissue into the blood, which usually includes lactate dehydrogenase (LDH), BNP, cardiac troponin I (cTn-I), and creatine kinase myoglobin (CK-MB) [32]. The SGI treatments attenuated the upregulation of serum BNP, CK-MB, cTn-I concentrations, and LDH activity stimulated by ischemia-reperfusion (Figure S2a–d, g). Considering oxidative stress contributes to the pathogenesis of MIR injury, we measured the changes of oxidative stress-associated marker molecules including malondialdehyde (MDA) and superoxide dismutase (SOD) upon SGI treatment. The results showed that SGI downregulated the MDA level and upregulated the SOD activity both in the serum and in the myocardial tissue (Figure S2e-f, h-i), suggesting that SGI attenuated the oxidative stress under MIR condition [33–35].

The article "Salviae miltiorrhizae Liguspyragine Hydrochloride and Glucose Injection Protects against Myocardial Ischemia-Reperfusion Injury and Heart Failure" was retracted in 2023. Reasons: signs of a paper mill; suspected computer-generated content; unreliable results or conclusions; concerns about the data.

### 3.2. SGI Improves Cardiac Function in Zebrafish Induced by H/R

A zebrafish larvae hypoxia/reoxygenation (H/R) model has been established to simulate MIR [36]. Here, we utilized this zebrafish H/R model to further study the role of SGI in MIR injury. Firstly, we titrated the SGI concentration in fish by analyzing its effects on the livability, heart rate, and gross morphology of zebrafish embryos. SGI at 0.025 mg/ml showed no effect on those characteristics and was selected for follow-up studies (Figure S3a-c). Under H/R stimulation, the heart rate of zebrafish embryos decreased significantly, and the SV, EF, FAC, and CO all decreased obviously, and the SGI treatment restored those characteristics to a level close to control fish without H/R stimulation (Figure S4a-e). Those results indicated that SGI can improve the cardiac impairment of zebrafish induced by H/R.

### 3.3. The Protective Effect of SGI on H9c2 Cardiomyocytes Induced by H/R

After demonstrating a protective role of SGI on MIR injury with the rat and zebrafish models, we further consolidated those findings by using a cardiomyocyte H/R model. The survival rates of H9c2 cardiomyocytes at H/R time of 2-2 h, 2-4 h, 2-6 h, 4-4 h, and 6-6 h were significantly lower than that of the control group in a time-dependent manner (Figure S5a), and 4 h hypoxia-4 h reoxygenation (survival rate of 57.87%) was selected as the modeling conditions. For the SGI dosage titration, SGI at 0.048-480 *μ*M showed no inhibitory effect on the survival rate of H9c2 cardiomyocytes and thus was selected for subsequent experiments (Figure S5b). As shown in Figure S5c, SGI in the range of 0.48-480 *μ*M significantly increased the survival rate of H9c2 cardiomyocytes under the H/R condition. In addition, SGI can significantly increase the level of SOD (Figure S6a) and reduce the levels of LDH and MDA (Figure S6b, c) in the H9c2 cardiomyocytes, which is consistent with the above observation that SGI alleviated the oxidative stress in the rat MIR model.

### 3.4. SGI Attenuates the Activation of Autophagy under MIR Condition

Autophagy is massively activated during cardiac reperfusion, and therapeutic targeting of autophagy has shown beneficial effects under MIR condition. We further investigated whether SGI regulated the autophagy status in our rat MIR model. The results showed that ATG7, ATG5, Beclin1, and LC-3II/I expression levels in the model group were significantly increased, and SGI alleviated the overactivation of autophagy (Figure 2(a)). The regulatory effects of SGI on autophagy were further studied by detecting the changes in the expression or activation of autophagy regulators including JNK1, Bcl-2, mTOR, and Akt upon SGI treatment. We found that SGI treatment downregulated the p-JNK1 level while did not significantly affect the Bcl-2 level compared to the model group (Figure 2(b)). In addition, SGI inhibited the p-AKT and upregulated the p-mTOR level (Figure 2(c)). Those results suggested that SGI may alleviate the MIR injury via downregulating the activated autophagy under MIR conditions.

The article "Salviae miltiorrhizae Liguspyragine Hydrochloride and Glucose Injection Protects against Myocardial Ischemia-Reperfusion Injury and Heart Failure" was retracted in 2023. Reasons: signs of a paper mill; suspected computer-generated content; unreliable results or conclusions; concerns about the data.

Beclin1 and LC-3, as markers of autophagy, have become indicators of the degree of autophagy. Immunofluorescence staining was used to detect the localization of Beclin1 and LC-3 in the rat myocardial tissues, and the result showed that the expression levels of Beclin1 and LC-3 were significantly higher in the model group, while SGI significantly reduced the expression of Beclin1 and LC-3 (Figure S7a-b). This result further confirmed the inhibitory role of SGI in autophagy under MIR conditions.

Rapamycin (Rapa), as an autophagy inducer, caused a reduction of the survival rate of H9c2 cells in a dosage-dependent manner (Figure 2(d)). And SGI significantly improved the survival rate of H9c2 cells induced by Rapa (Figure 2(e)). Consistently, Rapa significantly deformed H9c2 cells, and 3-MA (autophagy inhibitor) and SGI significantly alleviated the deformation of H9c2 cells (Figure S7c).

### 3.5. SGI Improves Cardiac Function in Zebrafish Induced by ISO

ISO treatment in rats and zebrafish represents well-established heart failure models to investigate novel mechanisms and test new therapeutic strategies [37, 38]. In this study, we investigated whether SGI plays a protective role in ISO-induced heart failure. The ISO-induced myocardial injury resulted in an obvious decrease in heart rate accompanied by the formation of pericardium edema (Figures 3(a) and 3(b)), and in SV, EF, FAC, and CO as well. Zebrafish pericardium edema was relieved obviously upon SGI treatment, and the heart rate, SV, EF, FAC, and CO were all improved remarkably (Figures 3(c)–3(g)); these results indicated that SGI could improve the cardiac impairment of zebrafish induced by ISO.

Interestingly, we observed that ISO induced a shift of atrium-ventricle relative spatial position from top-bottom to a left-right pattern (Figure S8a), which may be caused by the formation of pericardial edema by ISO. And SGI restored the relative position of the ventricle and atrium to the normal (Figure S8a). In addition, SGI significantly inhibited the apoptosis of zebrafish cardiomyocytes induced by ISO treatment (Figure S8b).

The article "Salviae miltiorrhizae Liguspyragine Hydrochloride and Glucose Injection Protects against Myocardial Ischemia-Reperfusion Injury and Heart Failure" was retracted in 2023. Reasons: signs of a paper mill; suspected computer-generated content; unreliable results or conclusions; concerns about the data.

### 3.6. SGI Alleviates ISO-Induced Myocardial Injury in Zebrafish through Multiple Pathways

ISO has been previously proved to induce cardiac hypertrophy via increasing the expression of SP1, GATA4, ANP, BNP, and Prkg1a. In this study, we found that SGI significantly reduced the expression of these genes (Figures 4(a)–4(e)), suggesting that SGI can reduce the expression of ANP and BNP by inhibiting the SP1/GATA4 pathway, and playing a protective role on the heart. Furthermore, ISO was reported to activate autophagy by inhibiting Akt/mTOR [39], and SGI treatment significantly downregulated the mRNA expressions of ATG5, ATG7, LC-3, and Beclin1 (Figures 4(f)–4(i)), suggesting that SGI can play a protective role on zebrafish heart by inhibiting autophagy. In addition, SGI significantly reduced the expressions of *β* 1 adrenergic receptor (*β*1-AR), tyrosine hydroxylase 1 (Th1), and tyrosine hydroxylase 2 (Th2) mRNA (Figures 4(j)–4(l)), suggesting that SGI can play an antimyocardial injury effect by inhibiting the binding of ISO to *β*1-AR, inhibiting the expression of tyrosine hydroxylase, and reducing the production of catecholamine.

## 4. Discussion

SGI is being clinically used for occlusive cerebrovascular disease and other ischemic vascular diseases in China. Studies have shown that SGI has a protective effect on acute myocardial infarction induced by ISO in rats [40]. However, it is still unknown whether SGI plays therapeutic roles in other cardiovascular diseases including MIR injury and heart failure, and the underlying molecular mechanism of SGI acting on myocardial diseases remains a mystery. Here, we demonstrated that SGI protected against the MIR injury and heart failure by using in vivo rat and zebrafish MIR and heart failure models, and our preliminary mechanistic study showed that SGI may exert those effects via limiting the activation of the autophagy-related signal pathways and the natriuretic peptide pathway. When the heart is ischemic or hypoxic, aerobic oxidation of sugars is blocked, anaerobic glycolysis is enhanced, and permeability is elevated, leading to the release of various enzymes into the bloodstream, ultimately resulting in elevated levels of CK-MB, LDH, cTn-I, and BNP in serum or myocardial tissue [41]. The present study found that SGI could significantly reduce serum CK-MB, LDH, cTn-I, and BNP levels; NBT staining results also showed that the area of myocardial infarction in the SGI group was significantly reduced. This indicates that SGI has a better protective effect on MIR injury rats.

The article "Salviae miltiorrhizae Liguspyragine Hydrochloride and Glucose Injection Protects against Myocardial Ischemia-Reperfusion Injury and Heart Failure" was retracted in 2023. Reasons: signs of a paper mill; suspected computer-generated content; unreliable results or conclusions; concerns about the data.

Autophagy plays an important role in the heart, especially during MIR injury. In the reperfusion phase, autophagy over activates injured cells and even leads to cell death, thus negatively affecting the heart [42]. mTOR acts as a central regulator of physiology and pathology in the cardiovascular system by integrating intracellular and extracellular signals [43]. Both the mTOR-associated AMPK-mTOR pathway and the PI3K-Akt-mTOR pathway play an important role in MIR injury. During MIR injury, ATP stored in cardiomyocytes is rapidly depleted, and an increase in the adenosine monophosphate/adenosine triphosphate ratio rapidly activates AMPK energy receptors. Activated AMPK phosphorylates TSC2 [43], which in turn inhibits mTOR. Beclin1 was the first identified mammalian autophagy protein. After MIR injury, both Beclin1 protein levels and autophagy levels are upregulated [44]. The levels of autophagy and apoptosis caused by MIR were reduced after inhibition of Beclin1 expression by small-molecule interfering RNA technology at the in vitro level [45]. Immunofluorescence detection of Beclin1 and LC-3 performed in this study revealed high expression of Beclin1 and LC-3 in the myocardial tissue. Western blot analysis showed that SGI significantly downregulated the expression of ATG7, ATG5, and Beclin1 protein. Thus, our results indicate that autophagy occurred in rat myocardial tissue after MIR injury. The LC-3II/I ratio was significantly increased, suggesting that autophagy was overactivated. Simultaneously, we also found that SGI significantly upregulated the expression of mTOR and p-mTOR proteins and significantly downregulated the expression of p-JNK1 and p-AKT proteins. Those findings suggested that SGI may play an anti-MIR damage effect in rats by downregulating autophagy.

ANP and BNP are closely related to MIR, and ANP was shown to improve cardiac function by promoting the release of cGMP in isolated hypoxic reperfusion rat heart [46]. The ANP/PKG signaling pathway can regulate the K_ATP_ channel of ventricular cardiomyocytes [47]. ANP-modified adenosine oleate precursor drugs have a better therapeutic effect on acute myocardial ischemia in rats [48]. In this study, SGI significantly inhibited the expressions of ANP and BNP mRNA and significantly reduced the expressions of SP1 and GATA4 mRNA at the upstream and Prkg1a mRNA at the downstream, suggesting that SGI can play a protective role on the heart by inhibiting ANP and BNP. Both ISO and catecholamine can increase myocardial contractibility, heart rate, and oxygen consumption. However, a long-term increase in myocardial contractibility can lead to myocardial injury. Therefore, reducing the production of ISO and catecholamine or inhibiting their binding to their receptors can effectively treat myocardial injury. In this study, SGI significantly reduced the levels of *β*1-AR and TH mRNA, suggesting that SGI could reduce the binding of ISO to the receptor and reduce the generation of catecholamines by inhibiting TH expression.

The article "Salviae miltiorrhizae Liguspyragine Hydrochloride and Glucose Injection Protects against Myocardial Ischemia-Reperfusion Injury and Heart Failure" was retracted in 2023. Reasons: signs of a paper mill; suspected computer-generated content; unreliable results or conclusions; concerns about the data.

## 5. Conclusions

SGI has a protective effect on myocardial cell injury induced by H/R and Rapa. In addition, it can improve the cardiac function of zebrafish with H/R and ISO-induced injury, and the mechanism of action is related to inhibiting the expression of ANP and BNP, alleviating autophagy, reducing the binding between ISO and receptors, limiting the expression of TH, and reducing the generation of catecholamines. Furthermore, SGI protects cardiomyocytes by reducing oxidative stress and reducing the excessive release of CK and LDH. Meanwhile, the expression of Beclin1, ATG5, ATG7, and LC-3 autophagy proteins was downregulated through p-JNK1-Beclin1 and p-AKT-mTOR/p-mTOR-Beclin1 signaling pathways to rescue the cardiomyocyte from injury caused by excessive autophagy and to exert an anti-MIR injury effect.

## Figures and Tables

**Figure 1:** The protective effect of SGI on MIR in rats. (a, b) Dark blue represents normal myocardial tissue, and red represents infarcted myocardium. (c) The effect of SGI on heart rate. (d) The effect of SGI on the S-T segment. (e) Myocardial microstructure by transmission electron microscopy, red arrows represent myocardial fibers and yellow arrows represent mitochondria. Compared with the model group, ^∗^*P* < 0.05 and ^∗∗^*P* < 0.01.

**Figure 2:** SGI regulates the expression of autophagy-related proteins. (a) ATG7, Beclin1, ATG5, and LC-3II/I; (b) Bcl-2, JNK1, and p-JNK1; (c) Akt, p-Akt, mTOR, and p-mTOR; compared with the model group, ^∗^*P* < 0.05, ^∗∗^*P* < 0.01, and ^∗∗∗^*P* < 0.001. (d) The effect of different concentrations of Rapa on the survival rate of H9c2 cardiomyocytes, 80 *μ*M Rapa was selected to induce cardiomyocyte injury; (e) the effect of SGI on the survival rate of Rapa-induced H9c2 cardiomyocytes; compared with the control or Rapa group, ^∗∗∗^*P* < 0.001.

**Figure 3:** Improvement effect of SGI on heart function of ISO-induced zebrafish. Compared with the ISO group, ^∗∗^*P* < 0.01 and ^∗∗∗^*P* < 0.001.

**Figure 4:** SGI regulates the signal transduction of natriuretic peptide, autophagy, and ISO in zebrafish induced by ISO. Compared with the ISO group, ^∗^*P* < 0.05, ^∗∗^*P* < 0.01, and ^∗∗∗^*P* < 0.001.

The article "Salviae miltiorrhizae Liguspyragine Hydrochloride and Glucose Injection Protects against Myocardial Ischemia-Reperfusion Injury and Heart Failure" was retracted in 2023. Reasons: signs of a paper mill; suspected computer-generated content; unreliable results or conclusions; concerns about the data.

## Data Availability

The datasets generated during and/or analyzed during the current study are available from the corresponding author on reasonable request.

## Supplementary Materials

Supplementary Materials
Table S1 shows the information of reagents used in the experiment. Table S2 shows the gene primer sequences of zebrafish used for RT-PCR. Figure legends describe and explain supplementary Figures 1-8. In Methods: (1) How to establish a myocardial ischemia-reperfusion model in rats through surgery was introduced in detail. (2) Feeding and grouping of rats. (3) How to induce cardiac injury of zebrafish through hypoxia-reoxygenation and isoproterenol. (4) How to detect the cardiac function of zebrafish, including heart rate, cardiac volume, ejection fraction, cardiac output, and fractional area change. (5) Culture of cardiac myocytes. (6) RT-PCR detection of gene expression level in zebrafish, reagents, and corresponding article number. (7) Western blot was used to detect the protein expression level and specific operation steps in rat myocardial tissue. (8) The expression of LC-3 and Beclin1 proteins in rat myocardium was detected by immunofluorescence, and the specific procedures were followed. (9) Transmission electron microscopy (TEM) was used to observe the ultrastructure of rat myocardial tissue and the specific experimental methods.
